The article "Linc00210 drives Wnt/β-catenin signaling activation and liver tumor progression through CTNNBIP1-dependent manner" was retracted in 2022. Reasons: duplicated images; signs of a paper mill; original data or images not available; unreliable data.

# *Linc00210* drives Wnt/β-catenin signaling activation and liver tumor progression through CTNNBIP1-dependent manner

**DOI:** 10.1186/s12943-018-0783-3

**Published:** 2018-03-14

**Authors:** Xiaomin Fu, Xiaoyan Zhu, Fujun Qin, Yong Zhang, Jizhen Lin, Yuechao Ding, Zihe Yang, Yiman Shang, Li Wang, Qinxian Zhang, Quanli Gao

**Affiliations:** 1 Department of Cancer Biology Immunotherapy, The Affiliated Cancer Hospital of Zhengzhou University and Henan Cancer Hospital, 127 Dongming Road, Zhengzhou, Henan 450003 China; 2 Department of Histology and Embryology, College of Basic Medicine, Zhengzhou University, 100 Kexue Road, Zhengzhou, Henan 450052 China; 3 Department of Pathology, School of Medicine, University of Virginia, Charlottesville, VA 22908 USA; 4 Department of Otolaryngology, Medical School, University of Minnesota, Twin Cities Campus, Minneapolis, MN 55414 USA; 5 Department of Hepatopancreatobiliary Surgery, The Affiliated Cancer Hospital of Zhengzhou University and Henan Cancer Hospital, Zhengzhou, Henan 450003 China; 6 Department of Nuclear Medicine, The Affiliated Beijing Anzhen Hospital of Capital Medical University, Capital Medical University, Beijing, 100029 China

**Keywords:** *Linc00210*, CTNNBIP1, Wnt/β-catenin, Liver TICs, Copy number alterations

## Abstract

**Background:**

Liver tumor initiating cells (TICs) have self-renewal and differentiation properties, accounting for tumor initiation, metastasis and drug resistance. Long noncoding RNAs are involved in many physiological and pathological processes, including tumorigenesis. DNA copy number alterations (CNA) participate in tumor formation and progression, while the CNA of lncRNAs and their roles are largely unknown.

**Methods:**

LncRNA CNA was determined by microarray analyses, realtime PCR and DNA FISH. Liver TICs were enriched by surface marker CD133 and oncosphere formation. TIC self-renewal was analyzed by oncosphere formation, tumor initiation and propagation. CRISPRi and ASO were used for lncRNA loss of function. RNA pulldown, western blot and double FISH were used to identify the interaction between lncRNA and CTNNBIP1.

**Results:**

Using transcriptome microarray analysis, we identified a frequently amplified long noncoding RNA in liver cancer termed *linc00210*, which was highly expressed in liver cancer and liver TICs. *Linc00210* copy number gain is associated with its high expression in liver cancer and liver TICs. *Linc00210* promoted self-renewal and tumor initiating capacity of liver TICs through Wnt/β-catenin signaling. *Linc00210* interacted with CTNNBIP1 and blocked its inhibitory role in Wnt/β-catenin activation. *Linc00210* silencing cells showed enhanced interaction of β-catenin and CTNNBIP1, and impaired interaction of β-catenin and TCF/LEF components. We also confirmed *linc00210* copy number gain using primary hepatocellular carcinoma (HCC) samples, and found the correlation between *linc00210* CNA and Wnt/β-catenin activation. Of interest, *linc00210,* CTNNBIP1 and Wnt/β-catenin signaling targeting can efficiently inhibit tumor growth and progression, and liver TIC propagation.

**Conclusion:**

With copy-number gain in liver TICs, *linc00210* is highly expressed along with liver tumorigenesis. *Linc00210* drives the self-renewal and propagation of liver TICs through activating Wnt/β-catenin signaling. *Linc00210* interacts with CTNNBIP1 and blocks the combination between CTNNBIP1 and β-catenin, driving the activation of Wnt/β-catenin signaling. *Linc00210*-CTNNBIP1-Wnt/β-catenin axis can be targeted for liver TIC elimination.

## Background

Liver cancer is the third leading cause of cancer related death all over the world, and 90% liver cancers are hepatocellular carcinoma (HCC) [1]. Liver tumorigenesis is a complicated process, and the reason of tumorigenesis is still elusive. The tumor initiating cell model proposed that only a small subset cancer cells termed tumor initiating cells (TICs) account for tumor initiation, metastasis and recurrence [2]. TICs can self-renew and differentiate into various cells within tumor bulk [3]. Various surface markers have been found to identify and enrich liver TICs recently, including CD13, CD133, CD24, EPCAM and calcium channel α2δ1 [4–6]. While, the liver TIC biology remains largely unknown.

Several signaling pathways participate in liver cancer and liver TICs, including Wnt/β-catenin, Notch, Hedgehog and NF-κB signaling pathways [7]. Among these pathways, Wnt/β-catenin signaling is most widely investigated in tumor initiating cells and many adult progenitor cells, including intestinal stem cells, liver progenitor cells and so on [8, 9]. Wnt/β-catenin is also important for development, differentiation and many diseases, including various tumors [10]. As the core factor in Wnt/β-catenin signaling, β-catenin can form APC-β-catenin complex and β-catenin-TCF complex, accounting for its stability and activity, respectively [11]. CTNNBIP1, a β-catenin interacting protein, can block the binding of β-catenin and TCF/LEF, and thus functions as a negative regulator of Wnt/β-catenin activation [12]. As the importance of Wnt/β-catenin signaling in liver TICs, the regulatory mechanism of Wnt/β-catenin activation and the targeted therapy need further investigation.

As we know, many protein-coding genes participate in tumor formation and tumor initiation, including oncogenes and tumor suppresser genes [13]. Recently, long noncoding RNAs (LncRNAs) emerge as critical mediators in many biological processes. LncRNAs are defined as transcripts that are longer than 200 nucleotides (nt) without protein coding ability [14]. LncRNAs exert their roles through multi-layered regulation, including gene transcription, translocation, mRNA stability, protein stability, activity, subcellular location and so on. LncRNAs participate in gene expression by recruiting chromosome remodeling complex into gene promoter through trans- or cis- manners [14]. They also interact with some important proteins and regulate their stabilities or activities [15, 16]. LncRNAs play critical roles in many physiological and pathological processes, including self-renewal regulation and tumorigenesis [17, 18], however, the role of lncRNAs in liver TICs is largely unknown.

Compared with normal cells, cancerous cells have more frequent mutations and instable chromosomes [19]. Gene copy number alteration (CNA) and mutation are two common chromosome aberrances in tumor [20]. Gene CNA plays critical roles in tumor formation and progression [21–23]. Gene copy number alterations are related to gene expression. In liver cancer, the oncogenic signaling pathways (including Wnt/β-catenin) with high expression along with tumorigenesis are frequently copy-number gained, while, lowly expressed genes (including ARID1A and RPS6KA3) are copy-number deleted [21]. The expression levels of another well-known copy number gained gene, c-Myc, were also positively correlated to its copy number gain [24]. While, lncRNA copy number alteration and its role in liver cancer and liver TICs haven’t been reported. Here, we focused on lncRNAs located on Chromatin 1q, a frequent copy number gained region in liver cancer [25]. We analyzed transcriptome data of liver TICs and non-TICs, and found a copy number gained lncRNAs, termed *linc00210*, is highly expressed in liver cancer and liver TICs. *Linc00210* interacts with CTNNBIP1, blocks its inhibitory role for Wnt/β-catenin signaling, and thus drives the self-renewal of liver TICs.

## Results

### Copy number gain of *linc00210* in liver cancer

DNA copy number alteration is a driver of tumorigenesis, and many oncogenes have increased copy numbers in tumor cells, including c-Myc, FGFR, BCL2L1, DLC1, PRKC1, Sox2 and so on [26]. Copy number gain often accompanies with high expression of transcripts, and copy number deletion results decreased expression. Although gene CNA is deeply explored, whether lncRNA CNA occurs in tumorigenesis and its role remain unclear. For liver cancer, CNA of Chromatin 1q plays a critical role in tumorigenesis. To investigate the role of lncRNA CNA in liver tumorigenesis and liver TICs, we utilized online-available transcriptome dataset (GSE66529 [27]) and analyzed the expression levels of lncRNAs located on Chromatin 1q. From the 295 lncRNAs detected, many lncRNAs showed dysregulated expression levels in liver TICs (Fig. 1a). To explore these lncRNAs in liver TIC self-renewal, we selected 10 lncRNAs and silenced their expression in Hep3B and PLC with antisense oligos, and detected liver TIC self-renewal using sphere formation assay, a standard assay for TIC self-renewal. We found *linc00210* knockdown impaired the self-renewal of liver TICs (Fig. 1b). We then confirmed the CNA of *linc00210* using TCGA dataset, and found about 13% liver cancer samples have *linc00210* copy number gain (Fig. 1c). To further confirm the CNA of *linc00210* in liver cancer, we collected 72 HCC samples, extracted tumor DNA, and detected the copy number of *linc00210* using realtime PCR, and found 16 samples had copy number gain, including eleven 3-copy and five 4-copy samples (Fig. 1d). We also confirmed the realtime PCR results using DNA FISH (fluorescence in situ hybridization) (Fig. 1e).

**Fig. 1:** Copy number gain of *linc00210* in liver cancer. **a** Heat map of lncRNA expression levels in liver TICs and non-TICs. 295 lncRNAs located on Chromatin 1q were shown, and the top 50 highly expressed lncRNAs in liver TICs were listed in right. **b** Histogram of sphere formation ratios. Hep3B and PLC were transfected with the indicated antisense oligo, followed by sphere formation. 1000 cells were used for sphere formation assay. **c** *Linc00210* copy number analysis using TCGA datasets. *Linc00210* showed high frequency of copy number gain in breast cancer and liver cancer. **d** Realtime PCR confirmed the CNA of *linc00210*. 72 HCC DNA samples were extracted, and primers targeting *linc00210* DNA were used, primers targeting β-actin DNA were used for loading control. **e** *Linc00210* DNA FISH validated its copy number gain. According realtime PCR data of 1D, 2 copy samples, 3 copy samples and 4 copy samples were collected for *linc00210* DNA FISH. For each group, 5 samples were confirmed. Scale bars, 10 μm. **f** The relationship between *linc00210* copy number gain and *linc00210* transcript expression. Peri-tumor and HCC samples with 2, 3, 4 *linc00210* copy numbers were analyzed for *linc00210* expression. **g** Sphere formation assays were performed using *linc00210* copy number gained samples and control samples. Typical images were shown in left panels and scatter diagram were shown in right panels. Scale bars, 500 μm. **h** CD133^+^ TICs and CD133^−^ non-TICs were enriched by FACS and invasive capacity was examined by transwell assay. Typical images and cell numbers (mean ± s.d.) were shown. **i** Primary cells derived from HCC patients with *linc00210* 2 copies, 3 copies and 4 copies were examined for invasive capacity. Typical images and cell numbers (mean ± s.d.) were shown. 5 samples were examined for each group. *P < 0.05; **P < 0.01; ***P < 0.001 by two-tailed Student’s t test. Data are representative of three independent experiments

After confirming the CNA of *linc00210* in liver cancer, we also analyzed the relationship between *linc00210* CNA and expression levels, and found that higher expression levels in copy number gained samples (Fig. 1f). Meanwhile, we detected the sphere formation ability, and found *linc00210* copy number gained samples showed enhanced self-renewal capacity (Fig. 1g). Meanwhile, we confirmed that tumor initiating cells account for tumor invasion (Fig. 1h), and *linc00210* CNA is related to tumor invasion (Fig. 1i). Altogether, copy number gain of *linc00210* in liver cancer was correlated to *linc00210* expression and liver TIC self-renewal.

### *Linc00210* was highly expressed in liver cancer and liver TICs

We then examined the expression of *linc00210* in liver cancer and liver TICs. We detected *linc00210* expression using clinical samples, and found that *linc00210* was highly expressed in liver cancer, and the expression levels were associated with clinical severity (Fig. 2a, b). Of interest, if we focused on the ratios of *linc00210* highly expressed cells, we found *linc00210* was only highly expressed in a small subset cells in tumor bulk, both in early stage samples and advanced samples, especially in early stage samples (Fig. 2b). Through transcriptome data, we found *linc00210* is highly expressed in liver TICs (Fig. 1a), and thus we proposed that the rare *linc00210* highly expressed cells were liver TICs. Accordingly, we detected *linc00210* expression in liver TICs.

**Fig. 2:** High expression of *linc00210* in liver cancer and liver TICs. **a** Scatter diagram of *linc00210* expression in the indicated samples. RNA extracted from 19 peri-tumor, 7 early HCC samples and 12 advanced HCC samples was used for *linc00210* detection, *ACTB* served as loading control. **b** *Linc00210* expression and subcellular location in indicated samples were analyzed by in site hybridization (ISH). Typical images were shown in left panels and analyzed data were shown in right panels. Peri-tumor tissues, early HCC and advanced HCC tissues were used for *linc00210* staining. Because of different severity extent and heterogeneity between HCC samples, the staining looks very different. For every cell nucleus, *Linc00210* photon intensity > 100 were *Linc00210*^high^ cells. Three digoxin-labeled probes were used for linc00210 staining and their sequences were GCAAAAGGAAAAATCTGTTAG, TACCAGAAGGGCCTGTAAAG and CTCCTTCACCCTTATAAGCCT. **c**, **d** *Linc00210* expression levels in CD133^+^ liver TICs (**c**) and oncospheres (**d**) were analyzed using realtime PCR. Sample #1, #4 and #5 can form oncospheres in vitro and have CD133^+^ liver TICs. **e** *Linc00210* expression profiles in oncospheres were analyzed with fluorescence in situ hybridization (FISH) assays. c-Myc, a well-known liver TIC marker, was used as a control. Primary cells from sample #1 were used for sphere formation and staining. **f** Oncospheres were collected and nucleocytoplasmic segregation was performed. The nuclear and cytoplasmic fractions were used for RNA extraction, followed by realtime PCR for *linc00210* expression (left panels). The efficiency of nuclear cytoplasmic segregation was confirmed by Western blot (right panels). Sample #1, #4 and #5 were used for nucleocytoplasmic segregation. Scale bars, for B, 50 μm; for E, 10 μm. Throughout figure, data were shown as means±s.d. *P < 0.05; **P < 0.01; ***P < 0.001 by two-tailed Student’s t test. Data are representative of three independent experiments

We enriched liver TICs from primary samples using CD133, a widely-accepted liver TIC surface marker, and examined *linc00210* expression levels. Compared with CD133^−^ cells, CD133^+^ TICs showed elevated *linc00210* expression (Fig. 2c). Taking advantage of sphere formation assays, we collected oncospheres and non-spheres, examined *linc00210* expression, and also found *linc00210* was highly expressed in spheres (Fig. 2d). We also performed fluorescence in situ hybridization (FISH) using spheres and non-spheres, and confirmed the high expression of *linc00210* in oncospheres (Fig. 2e). Moreover, fluorescence results also indicated the nuclear location of *linc00210* (Fig. 2e). Nuclear-cytoplasmic segregation showed the consistent result with FISH (Fig. 2f). Altogether, *linc00210* was highly expressed in live cancer and liver TICs.

### *Linc00210* was required for liver TIC self-renewal

We next explored the role of *linc00210* in liver TIC self-renewal. Firstly, we established *linc00210* silenced cells using antisense oligos (Fig. 3a), and performed sphere formation assays. *Linc00210* knockdown impaired the sphere formation ability and CD133 expression, indicating its critical role in liver TIC self-renewal and maintenance (Fig. 3a, b). Sequential sphere formation assay also confirmed that *linc00210* participates in live TIC self-renewal (Fig. 3c). Using transwell assay, we also found *linc00210* was involved in tumor invasion (Fig. 3d).

**Fig. 3:** *Linc00210* was required for liver TIC self-renewal. **a** Impaired self-renewal of *linc00210* silenced cells. *Linc00210* were silenced with antisense oligo (ASO) (left panels), followed by sphere formation assays. Representative sphere images were shown in middle panels and calculated ratios were shown in right panels. For ASO transfection, 1 × 10^5^ primary cells were transfected with 0.7 μL jetPEI-Hepatocyte reagent (MBTR005, Himedia Company) containing 1 μg ASO. The transfection reagent was removed 24 h later and knockdown efficiency was examined 48 h later, followed by sphere formation. **b** Primary cells were treated with ASO and CD133 expression levels were examined by realtime PCR. Three samples were used and the mRNA levels were normalized to control cells. **c** Sequential sphere formation assays were performed using *linc00210* silenced and control spheres. Three samples were used. **d** *Linc00210* silenced and control cells were used for invasive capacity. Typical images and cell numbers (mean ± s.d.) were shown. **e** 1 × 10^6^ indicated cells were subcutaneously injected into BALB/c nude mice, and the established tumors were obtained one month later. Six mice were used for tumor propagation. **f**, **g** Tumor initiating capacities of the indicated cells were examined using gradient dilution xenograft model. 10, 1 × 10^2^, 1 × 10^3^, 1 × 10^4^, and 1 × 10^5^ *linc00210* silenced cells and control cells were subcutaneously injected into 6-week-old BALB/c nude mice. Tumor formation was observed 3 months later and the ratios of tumor-free mice were calculated (**f**). TIC ratios were calculated through extreme limiting dilution analysis (**g**). CI, Confidence interval; vs, versus. **h** *Linc00210* was transcriptionally repressed through CRISPRi strategy (left panels), followed by sphere formation. Typical images (middle panels) and calculated ratios (right panels) were shown. **i** Lnc00210 depleted cells were established through CRISPRi strategy and CD133 expression levels were examined by realtime PCR. Three samples were used and the mRNA levels were normalized to control cells. **j** 1 × 10^6^ *linc00210* silenced cells were subcutaneously injected into BALB/c nude mice, and the established tumors were obtained one month later. Six mice were used for tumor propagation. **k** *Linc00210* overexpressed cells were established (left panels), followed by sphere formation assay (middle and right panels). **l** CD133 expression levels in *lin00210* overexpressed and control cells were examined by realtime PCR. **m** Tumor propagation of *linc00210* overexpressed and control cells. 1 × 10^6^ indicated cells were used per mouse, and six mice were used for each group. **n**, **o** 10, 1 × 10^2^, 1 × 10^3^, 1 × 10^4^, and 1 × 10^5^ *linc00210* overexpressing cells and control cells were subcutaneously injected into 6-week-old BALB/c nude mice for tumor initiation. The ratios of tumor-free mice (**n**) and tumor initiating cells (**o**) were shown. CI, Confidence interval; vs, versus. For A, H, K, scale bars, 500 μm. Data were shown as means±s.d. **P < 0.01; ***P < 0.001 by two-tailed Student’s t test. Data are representative of three independent experiments

We then injected 1 × 10^6^ *linc00210* silenced cells into BALB/c nude mice, and found *linc00210* knockdown attenuated tumor propagation (Fig. 3e). To examine the tumor initiating capacity, 10, 1 × 10^2^, 1 × 10^3^, 1 × 10^4^ and 1 × 10^5^ cells were injected into BALB/c nude mice, and tumor formation was observed three months later. *Linc00210* depleted cells showed attenuated tumor initiating ability, confirming the critical role of *linc00210* in tumor initiation (Fig. 3f, g). To further confirm the role of linc00210 in liver TIC self-renewal, we established *linc00210* silenced cells using CRISPRi approach (Fig. 3h), followed by sphere formation, and found *linc00210* silenced cells showed impaired sphere formation capacity (Fig. 3h), maintenance (Fig. 3i) and tumor propagation (Fig. 3j).

We also constructed *linc00210* overexpressed primary cells, and detected their self-renewal capacity with sphere formation assays. *Linc00210* overexpression triggered more spheres and enhanced CD133 expression, confirming the promoting role of *linc00210* in liver TIC self-renewal and maintenance (Fig. 3k, l). On the contrary of *linc00210* silenced cells, *linc00210* overexpressed cells formed larger tumors, confirming the role of *linc00210* in tumor propagation (Fig. 3m). We also performed tumor initiation assay with *linc00210* overexpressed cells, showing enhanced tumor formation capacity (Fig. 3n) and increased TIC ratios (Fig. 3o) upon *linc00210* overexpression. Taken together, *linc00210* played an essential role in liver TIC self-renewal.

### *Linc00210* drove liver TIC self-renewal through Wnt/β-catenin signaling

To investigate the molecular mechanism of *linc00210* in liver TIC self-renewal, we detected the expression levels of target genes of self-renewal associated pathways (NFkB, Wnt/β-catenin, Notch and Hedgehog). *Linc00210* depleted cells showed decreased expression levels of Wnt/β-catenin target genes, while, other detected pathways weren’t influenced (Fig. 4a). To confirm the role of *linc00210* in Wnt/β-catenin activation, we transfected TOPFLash vector into *linc00210* silenced cells, followed by luciferase assay. The results showed impaired Wnt/β-catenin activation in *linc00210* knockdown cells, confirming the critical role of *linc00210* in Wnt/β-catenin signaling pathway (Fig. 4b). We then analyzed Wnt/β-catenin activation through Western blot, and also validated the critical role of *linc00210* in Wnt/β-catenin activation (Fig. 4c). Then we detected Wnt/β-catenin activation with *linc00210* overexpressed cells, and found enhanced Wnt/β-catenin activation upon *linc00210* overexpression, echoing the knockdown results (Fig. 4d, e). What is more, we detected the expression levels of Wnt/β-catenin target genes in *linc00210* copy number gained clinical samples, and found that Wnt/β-catenin was activated upon *linc00210* copy number gain (Fig. 4f, g). These data concluded that *linc00210* promoted Wnt/β-catenin activation.

**Fig. 4:** *Linc00210* participated in Wnt/β-catenin activation. **a** Heat map of indicated target genes in *linc00210* silenced and control cells. The target genes of Wnt/β-catenin signaling pathway (red genes) were decreased in *linc00210* silenced cells. **b** TOPFlash assay of *linc00210* silenced cells. TOPFlash and FOPFlash vectors were transfected into *linc00210* silenced cells and control cells, and luciferase intensity was detected 36 h later. **c** Western blot of Wnt/β-catenin target genes. *Linc00210* silenced and control cells were used for western blot. β-actin served as a loading control. The relative intensity was normalized to control (Ctrl) samples and shown below. **d** Heat map of target genes of self-renewal associated pathways. Wnt/β-catenin was activated upon *linc00210* overexpression. **e** Wnt/β-catenin activation in *linc00210* overexpressed cells was examined by Westen blot. **f**, **g** *Linc00210* copy number gained samples, non-gained samples and peri-tumor cells were analyzed for Wnt/β-catenin activation by detecting expression levels of target genes by realtime PCR (**f**) and Western blot (**g**). **h** Heat map of Wiki4 treated cells and control cells. **i** Self-renewal capacities of the indicated treated cells were analyzed using sphere formation assay. *Linc00210* was overexpressed in indicated treated and control cells, followed by sphere formation assays. Typical images were shown in upper panels and liver TIC ratios were shown in lower panels. **j** Wnt/β-catenin activation was inhibited in *linc00210* overexpressed and control cells, followed by transwell assay for invasive capacity. Typical images and cell numbers (mean ± s.d.) were shown. **k** The indicated Wnt/β-catenin targets were rescued in *linc00210* silenced cells, followed by sphere formation assay, and typical images were shown. Scale bars, 500 μm. Data were shown as means±s.d. **l** The indicated cells were used for transwell assay for invasive capacity and typical images were shown. Scale bars, 500 μm. For **a**, **d**, **h**, red represents high expression and blue represents low expression. **P < 0.01; ***P < 0.001 by two-tailed Student’s t test. Data are representative of three independent experiments

Considering that Wnt/β-catenin signaling is an important mediator for liver TIC self-renewal, and that *linc00210* participated in liver TIC self-renewal and Wnt/β-catenin signaling, we wanted to know whether *linc00210* drove liver TIC self-renewal through Wnt/β-catenin pathway. Accordingly, we inactivated Wnt/β-catenin signaling with Wiki4, a widely-used Wnt/β-catenin inhibitor (Fig. 4h), and overexpressed *linc00210*, followed by sphere formation. On the contrary of control cells, in Wiki4 treated cells, *linc00210* overexpression had no influence on liver TIC self-renewal, while, in other treated cells, *linc00210* overexpression could increase the sphere formation capacity (Fig. 4i). Using tumor invasion assay, we also confirmed *linc00210* promoted tumor invasion through Wnt/β-catenin signaling (Fig. 4j). To further confirm the role of Wnt/β-catenin signaling in *linc00210* mediated liver TIC self-renewal, we rescued three major Wnt/β-catenin targets in *linc00210* silenced cells and found spheres formation and invasion capacity were rescued (Fig. 4k, l). These results indicating that *linc00210* participated in liver TIC self-renewal through Wnt/β-catenin signaling.

### *Linc00210* interacted with CTNNBIP1

To further explore the mechanism of *linc00210* in Wnt/β-catenin activation and liver TIC self-renewal, we performed RNA pulldown assay, and detected the specific band in *linc00210* samples by mass spectrum. CTNNBIP1, an interacting protein of β-catenin, was detected in *linc00210* samples (Fig. 5a). We then confirmed the interaction between *linc00210* and CTNNBIP1 through RNA pulldown and western blot (Fig. 5b). We also performed mapping assay and found the third region (601–900 nt) of *linc00210* was required for its interaction with CTNNBIP1 (Fig. 5c). We overexpressed full-length and truncated linc00210 and found the third region was sufficient for Wnt/β-catenin activation (Fig. 5d). Additionally, taking advantage of this region as probe, we performed RNA electrophoretic mobility shift assay (RNA EMSA), and confirmed the interaction between *linc00210* and CTNNBIP1 (Fig. 5e). We also performed RNA immunoprecipitation, detected *linc00210* enrichment using realtime PCR, and found that *linc00210* was enriched in CTNNBIP1 samples (Fig. 5f). Finally, we observed the subcellular location of *linc00210* and CTNNBIP1 using RNA fluorescence in situ hybridization (RNA FISH). To large extent, *linc00210* and CTNNBIP1 were located together in primary samples (Fig. 5g), liver TICs and oncospheres (Fig. 5h), confirming the interaction between *linc00210* and CTNNBIP1. Altogether, *linc00210* interacted with CTNNBIP1 in liver TICs.

**Fig. 5:** *Linc00210* interacted with CTNNBIP1. **a** RNA pulldown assays were performed and samples were separated with SDS-PAGE and silver staining. *Linc00210* specific band was identified as CTNNBIP1 by Mass Spectrum. **b** The interaction between *linc00210* and CTNNBIP1 was confirmed by Western blot. Only *linc00210* can bind to CTNNBIP1. **c** The indicated regions of *linc00210* were constructed and their interaction with CTNNBIP1 was analyzed using RNA pulldown and Western blot assays. **d** *Linc00210* full length (FL) and the indicated truncates were overexpressed in sample #1 cells and the expression levels of *Axin2, MYC* and *TCF7* was examined by realtime PCR. **e** RNA electrophoretic mobility shift assay (RNA EMSA) was performed using *linc00210* region#3 and CTNNBIP1 proteins. CTNNBIP1 antibody was used for super shift. **f** RNA immunoprecipitation was performed using CTNNBIP1 antibody and control IgG, and the enrichments were analyzed using realtime PCR. Upper panels were fold enrichment and lower panels were gel results. ACTB served as a negative control. Data were shown as means±s.d. **g** HCC primary samples were stained with *linc00210* probes and CTNNBIP1 antibody, followed by observation with confocal microscope. **h** Co-localization of *linc00210* and CTNNBIP1 in liver TICs (upper panels) and oncospheres (lower panels). *Linc00210* probes and CTNNBIP1 antibody were used for staining. Scale bars, 20 μm. For G, H, three probes were labeled with digoxin for linc00210 staining and their sequences were GCAAAAGGAAAAATCTGTTAG, TACCAGAAGGGCCTGTAAAG and CTCCTTCACCCTTATAAGCCT. Data are representative of three independent experiments

### *Linc00210*-β-catenin signaling served as targets for liver TIC elimination

CTNNBIP1 interacts with β-catenin, inhibits the interaction between β-catenin and TCF/LEF complex, and thus blocks the activation of Wnt/β-catenin signaling. Here we found *linc00210* interacted with CTNNBIP1, next we wanted to explore the role of *linc00210* in β-catenin interactomics. Taking advantage of *linc00210* silenced cells, we performed immunoprecipitation using β-catenin antibody, and its interaction with CTNNBIP1, TCF3, TCF4 and LEF1 was examined using western blot. *Linc00210* knockdown cells showed enhanced CTNNBIP1-β-catenin interaction and impaired β-catenin-TCF/LEF interaction, indicating that *linc00210* inhibited CTNNBIP1-β-catenin interaction and drove Wnt/β-catenin activation through β-catenin-TCF/LEF complex (Fig. 6a). We also confirmed the role of *linc00210* in β-catenin interactomics using *linc00210* overexpressed cells (Fig. 6b). What is more, we examined the β-catenin interactomics using *linc00210* copy number gained samples, and found impaired CTNNBIP1-β-catenin interaction and enhanced β-catenin-TCF/LEF interaction upon *linc00210* copy number gain (Fig. 6c). Meanwhile, linc00210 didn’t participate in CTNNBIP1 expression (Fig. 6d) and the subcellular location of β-catenin (Fig. 6e). These data confirmed that *linc00210* promoted Wnt/β-catenin activation by blocking the inhibitory role of CTNNBIP1 and promoting the β-catenin-TCF/LEF interaction.

**Fig. 6:** *Linc00210*-Wnt/β-catenin signaling served as a target for liver TIC elimination. **a**-**c** β-catenin interaction analyses using co-immunoprecipitation assays with β-catenin antibody. *Linc00210* silenced cells (**a**), overexpression cells (**b**) and copy number gained samples (**c**) were crushed with RIPA lysis buffer, and incubated with β-catenin antibodies. The enrichment samples were analyzed using Western blot with the indicated antibodies. **d** CTNNBIP1 expression levels in *linc00210* silenced cells were examined by realtime PCR. **e** *Linc00210* silenced cells were performed with nucleocytoplasmic separation, and subcellular location of β-catenin was examined by Western blot. EEA1 and H3 were cytoplasmic and nuclear markers, respectively. **f** β-catenin knockout cells were established using CRISPR/Cas9 approach (left panels), followed by sphere formation assays for self-renewal analysis. Typical sphere images were shown in middle panels and liver TIC ratios were shown in right panels. **g** CD133 expression levels in β-catenin knockout cells were examined by realtime PCR. **h**, **i** CTNNBIP1 knockout cells were generated, followed by sphere formation (**h**) and CD133 examination (**i**). **j**, **k** Transwell assays were performed using β-catenin knockout (**j**) and CTNNBIP1 knockout (**k**) cells. Typical images and cell numbers (mean ± s.d.) were shown. **l** Liver TICs were injected into BALB/c nude mice, and tumors were treated with the indicated reagents every 2 days. One month later, tumors were collected and weighted. XAV-393 is an inhibitor for Wnt/β-catenin signaling. **m** The indicated treated tumors were collected and stained with CD133-PE, and CD133 positive cells were gated as shown. **n** Immunohistochemistry of with c-Myc using the indicated treated tumors. Scale bars, **f**, **h**, 500 μm; **n**, 50 μm. For **d**, **f**, **g**, **h**, **i**, **l**, data were shown as means±s.d. **P < 0.01; ***P < 0.001 by two-tailed Student’s t test. Data are representative of four independent experiments

We then investigated the role of β-catenin and CTNNBIP1 in liver TIC self-renewal. We established β-catenin knockout cells using CRISPR/Cas9 approach, followed by sphere formation assay. β-catenin knockout cells showed impaired self-renewal capacity and liver TIC maintenance (Fig. 6f, g). Similarly, CTNNBIP1 knockout cells were also generated through CRISPR/Cas9 approach, and showed enhanced self-renewal and maintenance of liver TICs (Fig. 6h, i). These data indicated that Wnt/β-catenin drove liver TIC self-renewal, and Wnt/β-catenin inhibitory protein CTNNBIP1 served as a negative regulator for liver TIC self-renewal. We also detected tumor invasion capacity and found β-catenin and CTNNBIP1 played opposite roles in tumor invasion regulation (Fig. 6j, k).

Finally, we detected whether *linc00210*-Wnt/β-catenin signaling could serve as targets in liver cancer and liver TIC elimination. We inhibited *linc00210* using antisense oligos, and inhibited Wnt/β-catenin signaling using Wiki4 and XAV-939. We found attenuate tumor propagation upon *linc00210*-Wnt/β-catenin inhibition (Fig. 6l). Taking advantage of the antibody against CD133, we detected the proportion of CD133^+^ liver TICs in tumor bulk, and found decreased liver TICs in *linc00210*-Wnt/β-catenin inhibited cells (Fig. 6m). We also detected c-Myc, another TIC self-renewal marker, using immunohistochemistry, and confirmed attenuate self-renewal of liver TICs upon *linc00210*-Wnt/β-catenin inhibition (Fig. 6n). Meanwhile, from the tissue morphology, we found control tumors were much more serious, with more heteromorphic nuclei (Fig. 6n). Altogether, *linc00210*-Wnt/β-catenin served as a target for liver cancer and liver TICs elimination.

## Discussion

Liver tumor initiating cells (TICs) are a small subset cells within tumor bulk that have self-renewal and differentiation capacity [28]. Tumor initiating cells have cancer property and stemness simultaneously [2, 29]. Several assays were established to examine liver TIC self-renewal, including surface markers, sphere formation, side population and diluted xenograft formation assay [30]. In this work, two widely accepted system, sphere formation in vitro and tumor initiation assay in vivo, were used to examine the self-renewal of liver TICs. Many stemness pathways are activated in liver TICs, including Wnt/β-catenin, Notch, Hedgehog, Yap1, and so on [31–33]. Other than signaling pathway, the key stemness factors, including Oct4, Sox2, Klf4 and c-Myc are also important for the self-renewal of liver TICs [30]. Based on transcriptome of liver TICs and non-TICs, here we identified a long noncoding RNA involved in liver TIC self-renewal, adding a new layer for Wnt/β-catenin activation and liver TIC self-renewal.

LncRNAs were considered as byproducts of RNA polymerase II, while, their important roles have been emerging these years [34]. LncRNAs regulate various physiological and pathological progresses, including tumorigenesis [34, 35]. LncRNAs participate in cancer proliferation, metastasis, drug resistance and energy metabolism [15, 17, 36–38]. Recently several papers discovered the critical role of lncRNAs in liver TIC self-renewal. Lnc β-Catm, a lncRNA highly expressed in liver TICs, interacts with β-catenin and promotes its stability through inhibiting its ubiquitination [33]. LncBRM interacts with BRM, and promotes the recruiting of BRG1 typed SWI/SNF to Yap1 promoter, and finally drives liver TIC self-renewal through Yap1 signaling [32]. LncSox4 binds to the Sox4 promoter and recruits SWI/SNF complex to facilitate Sox4 transcription [5]. Generally speaking, lncRNAs play critical roles in epigenetic regulation by recruiting various remodeling complexes to gene promoter, finally activating or inhibiting gene expression [27]. Recently several lncRNAs were also found to exert their roles through interacting with some important factors, including STAT3, P65, c-Myc and HIF1a [16, 37]. Here we found a CTNNBIP1 interacting lncRNA. By interacting with CTNNBIP1, *linc00210* blocks the inhibitory role of CTNNBIP1 in Wnt/β-catenin activation, and enhances the interaction of β-catenin and TCF/LEF complex, and finally drives Wnt/β-catenin signaling pathway activation. Actually, several lncRNAs were found to participate in Wnt/β-catenin activation, including *lncTCF7* [27], *lnc β-Catm* [33] and *lncRNA-LALR1* [39]. Mechanically, *lncTCF7* recruits NURF complex to TCF7 promoter to activate Wnt/β-catenin signaling [27]; *lnc β-Catm* binds to and stabilizes β-catenin directly [33]; lncRNA-LALR1 recruits CTCF [39] to Axin1 promoter, suppresses its expression and thus drives Wnt/β-catenin activation. Here, we found another Wnt/β-catenin regulator linc00210, which activates Wnt/β-catenin through an unreported mechanism.

*Linc00210* is highly expressed in liver cancer, with frequent CNA. Many genes, especially oncogenes, gained more copy numbers along with tumorigenesis; while, lincRNA copy number gain is rare reported. PVT1, a long noncoding RNA near from c-Myc loci, has copy number gain in breast cancer, and plays a critical role in tumorigenesis [24]. Here we focused on lncRNA copy number and found gained copy number of *linc00210* in liver TICs. *Linc00210* copy number gain is related to increased *linc00210* expression, activated Wnt/β-catenin signaling and enhanced liver TIC self-renewal. Of note, we found only 16 samples with copy number gain in 72 samples examined. Actually, 22.2% (16/72) is a relatively high frequency of copy number gain (compared to c-Myc CNA fraction [24]). Through realtime PCR and Western blot, we confirmed the correlation between linc00210 CNA and expression. Using molecular and cellular methods, we found *linc00210* promoted Wnt/β-catenin signaling through CTNNBIP1. *Linc00210* blocked the inhibitory role of CTNNBIP1, promoted the interaction between β-catenin and TCF/LEF complex, and finally activated Wnt/β-catenin signaling. Our results discovered a rare mechanism for Wnt/β-catenin activation and subsequent liver TIC self-renewal.

Wnt/β-catenin signaling, the key mediator for TIC self-renewal, plays a critical role in development, stemness and disease [10, 40–42]. There are many regulation mechanisms of β-catenin. For instance, APC degradation complex and β-catenin-TCF activating complex regulate β-catenin stability and activation, respectively [43]. Here, we reported a novel regulatory mechanism of Wnt/β-catenin activation. What is more, a copy number amplified long noncoding RNA *linc00210* is required for Wnt/β-catenin activation. Using sphere formation assay, tumor propagation and tumor initiation, we proved that targeting *linc00210*-Wnt/β-catenin signaling was an efficient way to eliminate liver cancer and liver TICs, providing a new avenue for liver TIC targeting. Here we found linc00210 interacted CTNNBIP1 to modulate β-catenin activation. However, in linc00210 non-gained samples, the activation of Wnt/β-catenin can also be modulated and participate in tumorigenesis, indicating other regulatory mechanisms in Wnt/β-catenin activation (for example, increased expression of bipartite complex partner of β-catenin or TCFs) also exist. The relationship between linc00210 and other Wnt/β-catenin modulators remains further investigation.

Above all, copy number gain of long noncoding RNA *linc00210* is related to high expression of *linc00210*, which blocks the interaction of β-catenin and CTNNBIP1. The impaired CTNNBIP1-β-catenin interaction promotes β-catenin-TCF/LEF interaction, and finally drives the activation of Wnt/β-catenin signaling and liver TIC self-renewal. *Linc00210* copy number gain, *linc00210* expression levels, CTNNBIP1 and β-catenin interaction are related to clinical severity of liver cancer and liver TIC self-renewal, which can be served as targets for eradicating liver TICs.

## Methods

### Cells and samples

293 T cells (ATCC CRL-3216), liver cancer cell line Hep3B (ATCC HB-8064) and PLC (ATCC CRL-8024) were obtained from ATCC. Cells were maintained in DMEM medium, supplemented with 10% FBS (Invitrogen), 100 μg/ml penicillin, and 100 U/ml streptomycin.

Human liver cancer specimens were obtained from the department of hepatopancreatobiliary surgery, with informed consent, according to the Institutional Review Board approval. All experiments, involving human sample and mice, were approved by the institutional committee of Henan Cancer Hospital. Sample #1: advanced hepatocellular carcinoma, 57 years old, male, tumor size, 7.5 × 6.2 × 4.7 mm, non-metastasis. Sample #4: advanced hepatocellular carcinoma, 68 years old, male, tumor size, 8.6 × 7.3 × 5.2 mm, metastasis. Sample #5: advanced hepatocellular carcinoma, 63 years old, female, tumor size, 6.6 × 5.9 × 5.2 mm, non-metastasis. Sample #1 had 3 copies of linc00210 and relative high linc00210 expression, sample #4 and #5 modestly expressed linc00210 with 2 copy numbers.

### Antibodies and reagents

Anti-β-actin (cat. no. A1978) were purchased from Sigma-Aldrich. Anti-β-catenin (cat. no. ab32572), anti-CTNNBIP1 (cat. no. ab129011) antibodies were from Abcam. Anti-histone H3 (cat. no. 4499), anti-Axin2 (cat. no. 5863), anti-TCF3 (cat. no. 2883), anti-TCF4 (cat. no. 2565), anti-LEF (cat. no. 2286), anti-TCF7 (cat. no. 2203) antibodies were from Cell Signaling Technology. Phycoerythrin (PE)-conjugated CD133 (cat. no. 130098826) was from MiltenyiBiotec. Anti-EEA1 (sc-53,939), anti-Myc (sc-4084) antibodies were purchased from Santa Cruz Biotechnology. Alexa594-conjugated donkey anti-rabbit IgG (cat. no. R37119) and Alexa488-conjugated donkey anti-mouse IgG (cat. no. R37114) antibodies were from Molecular Probes, Life Technologies. DAPI (cat. no. 28718–90-3) were obtained from Sigma-Aldrich. T7 RNA polymerase (cat. no. 10881767001) and Biotin RNA Labeling Mix (cat. no. 11685597910) were purchased from Roche Life Science. The LightShift Chemiluminescent RNA EMSA kit (cat. no. 20158) and Chemiluminescent Nucleic Acid Detection Module (cat. no. 89880) were from Thermo Scientific.

### TOPFlash luciferase assay

Wnt/β-catenin TOPFlash reporter (Addgene, 12,456) and mutant FOPFlash reporter (Addgene, 12,457) were transfected into indicated cells, along with thymidine kinase (TK), antisense oligo or control oligo. 36 h later, cells were lysed and detected with dual-detection luciferase detection kit (Promega Corporation, cat. no. E1910). Wnt/β-catenin activation was measured according to the fold change of TOPFlash versus the FOPFlash control.

### Sphere formation

For sphere formation assay, proper cells were seeded in Ultra Low Attachment 6-well plates and cultured in DMEM/F12 (Life Technologies) supplemented with B27, N2, 20 ng/ml EGF and 20 ng/ml bFGF. The spheres were counted and sphere pictures were taken 2 weeks later. For sphere formation assay, 1000 HCC cell line (Hep3B, PLC) cells or 5000 primary cells were used. bFGF (cat. no. GF446-50UG) was purchased from Millipore. EGF (cat. no. E5036-200UG), N2 supplement (cat. no. 17502–048) and B27 (cat. no. 17504–044) were from Life Technologies. Ultra low attachment plates (cat. no. 3471) were purchased from Corning Company.

Two weeks later, we collected medium containing spheres and non-sphere cells into an eppendorf tube and let stand for 5 min for sphere/non-sphere separation. The pellets were spheres, and supernatants were non-sphere cells. Supernatants were removed into a new eppendorf tube and collected by centrifugation at 4000 rpm for 5 min. Spheres and non-spheres were derived from the same cell lines or primary samples.

### Transwell invasion assay

For transwell invasion assays, 3 × 10^5^ HCC primary cells were plated onto the top chamber with Matrigel-coated membrane, and incubated in FBS-free medium. FBS containing medium was added in the lower chamber as a chemoattractant. The plate was incubated in incubator for 36 h and cells that did invade through the membrane were removed by a cotton swab, and the cells on the lower surface of the membrane were fixed with methanol and stained with crystal violet. The images were taken with Nikon-EclipseTi microscopy.

### Nucleocytoplasmic separation

5 × 10^6^ oncosphere cells were resuspended in 0.5 ml resuspension buffer (10 mM HEPES, 1.5 mM MgCl2, 10 mM KCl, 0.2% N-octylglucoside, Protease inhibitor cocktail, RNase inhibitor, pH 7.9) for 10 min’s incubation, followed by homogenization. The cytoplasmic fraction was the supernatant after centrifugation (400 g × 15 min). The pellet was resuspended in 0.2 ml PBS, 0.2 ml nuclear isolation buffer (40 mM Tris-HCl, 20 mM MgCl2, 4% Triton X-100, 1.28 M sucrose, pH 7.5) and 0.2 ml RNase-free H2O, followed by 20 min’s incubation on ice to clean out the residual cytoplasmic faction. The pellet was nuclear fraction after centrifugation. RNA was extracted from nuclear and cytoplasmic fractions using RNA extraction kit (Tiangen Company, Beijing). *Linc00210* content was examined by real-time PCR (ABI7300).

For *Linc00210* content, standard reverse transcription was performed using reverse transcription kit (Promega). Notably, same amount of RNA and same volume of cDNA were required. In our experiment, 1 μg nuclear RNA and 1 μg cytoplasmic RNA were used, with the same final volume of nuclear and cytoplasmic cDNA (50 μl). Real-time PCR was performed using 1 μl nuclear cDNA or 1 μl cytoplasmic cDNA, with the same primers and ABI7300 profile. The relative *Linc00210* contents were calculated using these formulas: nuclear ratio = 2^-Ct(nuclear)^ / (2^-Ct(nuclear)^ + 2^-Ct(cytoplasmic)^); cytoplasmic ratio = 2^-Ct(cytoplasmic)^ / (2^-Ct(nuclear)^ + 2^-Ct(cytoplasmic)^).

### Immunohistochemistry

Formalin-fixed liver cancer sections were deparaffinized in xylene and rehydrated in graded alcohols. After treated in 3% Hydrogen Peroxide (H_2_O_2_), the slides were incubated in boiled Tris-EDTA buffer (10 mM, pH 8.0) for antigen retrieval. Then the sections were incubated in primary antibodies and subsequent HRP-conjugated secondary antibodies. After detection with standard substrate detection of HRP, the sections were stained with hematoxylin and dehydration in graded alcohols and xylene.

### Tumor propagation and initiating assay

For tumor propagation, 1 × 10^6^ *linc00210* silenced, overexpressed and control cells were subcutaneously injected into 6-week-old BALB/c nude mice. After 1 month, the mice were sacrificed and tumors were obtained for weight detection. For every sample, 6 mice were used.

For tumor initiating assays, 10, 1 × 10^2^, 1 × 10^3^, 1 × 10^4^, and 1 × 10^5^ *linc00210* silenced cells were subcutaneously injected into 6-week-old BALB/c nude mice. Tumor formation was observed 3 months later, and the ratios of tumor-free mice were shown. Tumour-initiating cell frequency was calculated using extreme limiting dilution analysis [44] and an online-available tool (http://bioinf.wehi.edu.au/software/elda/). For every samples, 6 mice were used.

### CRISPRi depletion system

For Linc00210 depletion, dCas9-Krab CRISPRi strategy was used [45]. Briefly, dCas9 conjugated Krab (transcription repressor) was constructed for Linc00210 transcriptional inhibition. sgRNA was generated by online-available tool (http://crispr.mit.edu/) and lentivirus was generated in 293 T cells.

### *Linc00210* overexpression

*Linc00210* overexpressed cells was generated as described [27]. Briefly, full-length *linc00210* cDNA was cloned into pCDNA3.1 vector, and transfected cells with jetPEI-Hepatocyte reagent. Stable clones were obtained by selection with G418. All constructs were confirmed by DNA sequencing.

### Coimmunoprecipitation and RNA immunoprecipitation

For coimmunoprecipitation, *linc00210* silenced or copy number gained samples were crushed in RIPA buffer, followed by a 4-h’ incubation with β-catenin antibody. The precipitate was detected with Western blot.

For RIP, oncospheres were treated with 1% formaldehyde for crosslinking, and then crushed with RNase-free RIPA buffer supplemented with protease-inhibitor cocktail and RNase inhibitor (Roche). The Supernatants were incubated with CTNNBIP1 or control IgG antibodies and then Protein AG beads. Total RNA was extracted from the eluent, and *linc00210* or control ACTB enrichment was detected using real-time PCR.

### Statistical analysis

Two-tailed Student’s t tests were used for statistical analysis. *P* < 0.05 was considered to be statistically significant.

## Conclusion

In conclusion, this study defined a copy number gained lncRNA linc00210 in liver tumorigenesis and live TICs. With high expression in liver cancer and liver TICs, linc00210 was required for the self-renewal of liver TICs. Moreover, we found linc00210 interacted with CTNNBIP1 and modulated the activation of Wnt/β-catenin signaling. Linc00210-Wnt/β-catenin signaling can be targeted for liver TICs elimination. These findings revealed lncRNA copy number gain may be therapeutic target against liver TICs.
